# The Wnt/*β*-Catenin Pathway Regulated Cytokines for Pathological Neuropathic Pain in Chronic Compression of Dorsal Root Ganglion Model

**DOI:** 10.1155/2021/6680192

**Published:** 2021-04-19

**Authors:** Ye Zhang, Dan Zhao, Xutong Li, Beiyao Gao, Chengcheng Sun, Shaoting Zhou, Yanhong Ma, Xuemei Chen, Dongsheng Xu

**Affiliations:** ^1^Department of Rehabilitation, Shanghai Jiaotong University Affiliated Sixth People's Hospital, Shanghai 200233, China; ^2^Rehabilitation Section, Spine Surgery Division of Department of Orthopedics, Tongji Hospital Affiliated to Tongji University School of Medicine, Shanghai 200065, China; ^3^Department of Neurology, Minhang Hospital Affiliated to Fudan University, Shanghai 201100, China; ^4^Department of Rehabilitation Medicine, China-Japan Friendship Hospital, Beijing 100029, China; ^5^Department of Anatomy, College of Basic Medicine Sciences, Zhengzhou University, Zhengzhou, Henan 450001, China; ^6^Department of Rehabilitation Medicine, Yueyang Hospital of Integrated Traditional Chinese and Western Medicine, Shanghai 200437, China; ^7^School of Rehabilitation Science, Shanghai University of Traditional Chinese Medicine, Shanghai 201203, China; ^8^Engineering Research Center of Traditional Chinese Medicine Intelligent Rehabilitation, Ministry of Education, Shanghai 201203, China

## Abstract

Neuropathic pain is one of the important challenges in the clinic. Although a lot of research has been done on neuropathic pain (NP), the molecular mechanism is still elusive. We aimed to investigate whether the Wnt/*β*-catenin pathway was involved in NP caused by sustaining dorsal root ganglion (DRG) compression with the chronic compression of dorsal root ganglion model (CCD). Our RNA sequencing results showed that several genes related to the Wnt pathway have changed in DRG and spinal cord dorsal horn (SCDH) after CCD surgery. Therefore, we detected the activation of the Wnt/*β*-catenin pathway in DRG and SCDH and found active *β*-catenin significantly upregulated in DRG and SCDH 1 day after CCD surgery and peaked on days 7-14. Immunofluorescence results also confirmed nuclear translocalization of active *β*-catenin in DRG and SCDH. Additionally, rats had obvious mechanical induced pain after CCD surgery and the pain was significantly alleviated after the application of the Wnt/*β*-catenin pathway inhibitor XAV939. Furthermore, we found that the levels of proinflammatory factors tumor necrosis factor-*α* (TNF-*α*) and interleukin-18 (IL-18) were significantly elevated in CCD rat serum, while the levels of them were correspondingly decreased after the Wnt/*β*-catenin pathway being inhibited. The results of Spearman correlation coefficient analysis showed that the levels of TNF-*α* and IL-18 were negatively correlated with the mechanical withdrawal thresholds (MWT) after CCD surgery. Collectively, our findings suggest that the Wnt/*β*-catenin pathway plays a critical role in the pathogenesis of NP and may be an effective target for the treatment of NP.

## 1. Introduction

Low back pain (LBP) is the most common of all chronic pain disorders, and 80% of people experience LBP in their lifetime. LBP is often caused by lumbar foraminal stenosis (LFS) and lumbar disc herniation (LDH), causing symptoms such as motor dysfunction and NP [1]. In most parts of the world, LBP has become the main reason for limited mobility and job loss, which brings a huge economic burden to individuals, families, and society [2, 3]. Despite decades of investigation and tremendous research effort in NP, the specific cellular and molecular mechanisms remain elusive. From previous studies, we know many processes participated in the production and persistence of NP, including hyperexcitability of neurons due to changes in ion channels on neuronal membrane such as sodium channels [4], calcium channels [5], potassium channels [6, 7], inflammatory factor accumulation [8, 9], and activation of glial cells [10–12].

The Wnt/*β*-catenin pathway is one of three Wnt pathways, and active *β*-catenin is the key protein on the Wnt/*β*-catenin pathway. In the absence of Wnts, the destruction complex which is located in the cytoplasm will bind active *β*-catenin and phosphorylate it to inactive *β*-catenin and after that proteasome will degrade *β*-catenin. While Wnts bind Frizzled (Fzd) and LRP5/6 on the cell membrane, the destruction complex will subsequently disintegrate, and then, active *β*-catenin is not phosphorylated and accumulates in the cytoplasm, subsequently translocating into the nucleus, in which active *β*-catenin interacts with T cell/lymphoid enhancer factor (TCF/LEF) transcription factors, resulting in the target gene transcription such as TNF-*α* and IL-18 [13–15]. Recent studies have found that conditional deletion of one copy of Wntless or *β*-catenin through Nestin-Cre-mediated recombination was sufficient to suppress the expression of brain-derived neurotrophic factor (BDNF), a major neurotrophic factor in mammals [16, 17]. Besides, several studies revealed the Wnt pathway plays an important role in the production and persistence of NP, such as partial sciatic nerve ligation (PSL) [18], spinal nerve ligation (SNL) [19], and chronic constriction injury (CCI) [15]. However, the role of this pathway has not been reported in the CCD model, which is the ideal model for studying this pain because it is a realistic model that mimics the pathological changes and clinical symptoms of LBP [20]. Based on the above research basis, we put forward a hypothesis about the Wnt/*β*-catenin pathway may make an important impact on the pathogenesis of NP induced by CCD.

In our research, we first found that several genes related to the Wnt pathway have undergone significant changes through RNA sequencing analysis, and then, we investigated the role of the Wnt/*β*-catenin pathway in the generation and persistence of NP using the CCD model which is a well-characterized rat model. The CCD model is divided into a single nerve root compression model and two nerve roots' compression model. In this study, we chose the L4 and L5 nerve roots' compression model, because clinically, most of the LFS and LBP produce compression on multiple nerve roots instead of a single nerve root [21], so L4 and L5 nerve roots' compression can better simulate the actual clinical situation. We first studied the activation of the Wnt/*β*-catenin pathway over time in DRG and SCDH after CCD-induced NP. After that, we inhibited the activation of the Wnt/*β*-catenin pathway in DRG and SCDH through using XAV939, a small molecule tankyrase inhibitor which targets the Wnt/*β*-catenin pathway and inhibits the abnormal activation of the Wnt/*β*-catenin pathway without affecting normal function of cells [22], to observe if CCD-induced noxious hypersensitivity can be alleviated. XAV939 has good plasma stability and can be administered by intraperitoneal injection, which is more convenient than other Wnt pathway inhibitors [23]. Finally, we explored the potential mechanism of Wnt/*β*-catenin signaling in the generation and persistence of NP.

## 2. Experimental Procedures

### 2.1. Animals

Fifty-nine SD (Sprague Dawley) male rats (220 g-250 g body weight) were purchased from Shanghai Jiesijie Experimental Animal Co., Ltd (Shanghai, China, license no. SCXK (Hu) 2018-0004). Animals were housed in padded cages at a constant temperature (12 : 12 h light-dark cycle) and got food irradiated by the standard laboratory (Shanghai Jiesijie Experimental Animal Co., Ltd, China) and tap water with freedom. The animal experiments and handlings were approved by the Animal Ethics Committee of Tongji Hospital, Shanghai.

### 2.2. CCD Surgery

To produce intervertebral foramen stenosis and NP, the CCD model was used. The procedure for CCD has been described [24], and the schematic diagram of CCD is shown in Figure 1(a). Briefly, under 1% sodium pentobarbital anesthesia (0.4 ml/kg, i.p.) and sterile conditions, the left L4 and L5 intervertebral foramina of the rat were exposed, and then, two L-shaped stainless steel rods with a diameter of 0.6 mm and a length of 4 mm were inserted into the two intervertebral foramina, respectively, to produce chronic compression on the DRG. Finally, rats were kept in a single plastic cage after suturing muscle and skin. As for the sham group, the procedure is the same as that of the CCD group above but without the insertion of stainless steel rods [24]. During the experiment, no death or self-harm occurred in the rats. On the first postoperative day, rats with insignificant pain behavior were excluded (no positive response at 6 g).

### 2.3. Pharmacological Inhibition of the Wnt/*β*-Catenin Pathway

XAV939, an inhibitor of the Wnt/*β*-catenin pathway (Abmole, USA), in 10% DMSO/90% 0.9% NaCl, was injected in doses of 1.25 mg/kg intraperitoneal. Besides, the sham+vehicle group and the CCD+vehicle group also received an injection (200 *μ*l of 10% DMSO/90% 0.9% NaCl). The injections above were given at about 10 am every day for seven consecutive days.

### 2.4. Assessment of MWT

The rats were placed in a transparent box on the test grid at 8 am on test day, maintained at 25°C at room temperature, and adapted to the environment for 15-30 min. Von Frey hairs (Stoelting, USA) were applied, according to former reports [25], and the Von Frey hair number was selected as described [26], in brief, starting from 0.6 g, gradually increasing 1.0 g, 1.4 g, 2.0 g, 4.0 g, 6.0 g, 8.0 g, 10.0 g, 15.0 g, and 26.0 g. The sole of the hind paw was the site of stimulation of Von Frey hair, and the testing was performed only on the ipsilateral side. If the response was positive, the adjacent decreasing Von Frey hair was selected for the next stimulation; if the response was negative, the adjacent increasing hair was selected. The assessment was over when the maximum number of grams of 26.0 g was used and the response was still negative, or the test was performed three times after the first positive reaction. The MWT was calculated by the analyzer who was blind to the group data.

### 2.5. RNA Sequencing and Differentially Expressed Gene (DEG) Screening

Rats were anesthetized with 2% pentobarbital sodium (80 mg/kg) by intraperitoneal injection 28 days after CCD and decapitated after reaching full anesthesia. The left L4 and L5 nerves were quickly exposed and were carefully extracted. Then, the enlarged DRG was cut with a blade on ice. Later, according to the positioning of the lumbar enlargement, the dorsal horn of the left spinal cord of L4-5 segment was removed. All the tissues above were, respectively, placed in centrifuge tubes containing RNA later (QIAGEN, Valencia, CA) and were subsequently transferred to a 4°C refrigerator. RNA sequencing was completed by Shanghai Genergy Biotechnology Company, and the general protocol was as follows: 1 *μ*l RNA was taken for quantification and 500 ng RNA was taken for library construction according to the quantification results. After that, the library was subjected to quality inspection using Qubit instruments (Invitrogen, USA). Then, Illumina HiSeq was used for sequencing, and the instrument was NovaSeq 6000 (Illumina, USA). Deseq2 software (v1.16.1) was used to screen for DEGs, and the screening criteria are *P* value ≤ 0.05 and ∣log_2_ fold change | ≥1.

### 2.6. Western Blot Analysis

Rats were anesthetized with 2% pentobarbital sodium (80 mg/kg) by intraperitoneal injection and decapitated after reaching full anesthesia. The left L4-L5 DRG and SCDH segments were homogenized, respectively, by using the RIPA lysis buffer and then protein samples were quantified by applying BCA Protein Assay (Beyotime Biotechnology, Shanghai, China). The protein samples were separated by 10% SDS-PAGE (Beyotime Biotechnology, Shanghai, China) after being heated for 5 min at 99°C and subsequently transferred to 0.45 *μ*m PVDF membrane (Millipore, Billerica, MA). The membranes were treated with primary antibodies overnight at 4°C, after being blocked with 5% skimmed milk diluted in TBST, followed by being incubated in appropriate secondary antibodies. The following primary antibodies were used: rabbit anti-active *β*-catenin (1 : 1000 dilution; CST, Danvers, MA, USA), mouse anti-*β*-tubulin (1 : 1000 dilution; Sigma-Aldrich, Darmstadt, Germany), and horseradish peroxidase-linked secondary anti-rabbit or anti-mouse antibodies (1 : 1000 dilution; Beyotime Biotechnology, Shanghai, China). Finally, the blots were visualized by DRAFT-FluorChem Q (Alpha Innotech Corporation, San Leandro, CA, USA) and optical density of all bands was conducted by the ImageJ software (National Institutes of Health, Bethesda, MD, USA).

### 2.7. Immunohistochemistry

Rats were anesthetized with 1% pentobarbital sodium (40 mg/kg) by intraperitoneal injection. 0.9% saline and 4% paraformaldehyde were sequentially administered to these anesthetized rats. The L4 and L5 DRG were removed intact and subsequently fixed in 4% formaldehyde overnight. These tissues were then dehydrated with gradient sucrose (10%, 20%, and 30%) and frozen with OCT as they settled to the bottom in the 30% sucrose solution. After the embedding was completed, the tissues were sliced, and the thicknesses of the DRG and spinal cord sections were 10 *μ*m and 15 *μ*m, respectively. Next, immunofluorescence staining was performed, and the steps are as follows: after being blocked with a 0.01 M PBS blocking solution containing 10% goat serum and 0.3% Triton X-100 for 1 h at 37°C, the sections were incubated with the primary antibody overnight at 4°C (rabbit anti-active *β*-catenin, 1 : 800, Millipore), followed by being incubated in goat anti-rabbit Cy3-conjugated secondary antibody (1 : 300 dilution, Jackson ImmunoResearch, Amish, PA) for 2 hours at 37°C in the dark. Subsequently, sections were stained with nuclear dye DAPI (1 : 1000 dilution, Invitrogen, Carlsbad, CA, USA) for 7 minutes at 37°C in the dark. The sections were imaged with the confocal microscope (Nikon, A1 MP+, USA) and fluorescence microscope (Nikon, Ni-U, USA).

### 2.8. ELISA (Enzyme-Linked Immunosorbent Assay)

The rats in the deep anesthetized with sodium pentobarbital (80 mg/kg) were subjected to blood collection from the orbital venous plexus, and then, blood collected was centrifugated to get serum at 4000 rpm for 10 min at 4°C. Detailed steps were performed according to the kit (WESTANG BIO-TECH, Shanghai, China) instructions. The optical density (OD) value was measured by DENLEY DRAGON Wellscan MK 3 (Thermo Fisher Scientific, Waltham, MA, USA) at 450 nm, and all OD values were calculated after subtracting the blank value. Ascent software for Multiskan (Thermo Fisher Scientific, MA, USA) was applied to draw a standard curve, and the corresponding TNF-*α* and IL-18 concentrations were calculated according to the OD value of the sample.

### 2.9. Statistical Analysis

GraphPad Prism 7.0 software (GraphPad Software Inc., CA, USA) and SPSS 20.0 software (IBM Corporation, NY, USA) were applied to analyze all data. The number (*N*) of rats and the statistical significance were stated in the figures and figure legends. The sample size was determined based on previous experience. Two-way ANOVA was used to analyze the result of behavior, and one-way ANOVA was applied to analyze the western blot and ELISA. Spearman correlation coefficient analysis was used to analyze the correlation between MWT and inflammatory factor levels, including TNF-*α* and IL-18. Data are represented as mean ± SD (standard deviation). *P* < 0.05 was considered statistically significant.

## 3. Results

### 3.1. Induction and Persistence of Allodynia in CCD Model Rats

To confirm that the CCD model successfully and reproducibly induced tactile allodynia (Figure 1(a)), we performed gait and posture observations and measurements of MWT in CCD rats. We found that rats had gait and posture abnormalities after surgery, such as the hind paw of the operation side curled up and did not dare to bear weight. We tested the MWT of rats at different time points. The results showed that continuous compression of DRG significantly reduced the MWT of the hind paw and was consistent with previous studies [27, 28], as shown in Figure 1(b). The MWT decreased significantly on the first day after CCD and reached the lowest point on the 7th day (*P* < 0.0001). By the 28th day after surgery, the MWT remained at a low level (*P* < 0.0001). The MWT at each time point in the CCD group was lower than that in the sham group (*P* < 0.0001), while no obvious allodynia was observed in the sham group (*P* > 0.05).

### 3.2. Changes in the Expression of Wnt-Related Genes of DRG and SCDH in CCD

For selection of a subset of genes related to the Wnt pathway, the NCBI gene database and the Panther Classification System database system were used. “Wnt pathway” was used as a keyword to conduct a restrictive search for “rattus norvegicus.” 526 genes related to the Wnt pathway were obtained in the NCBI gene database. The overlapping genes of these data sets and the DEGs (differentially expressed genes) screened in the DRG and SCDH were analyzed using an online tool of the Venn diagram, and the results showed that 8 DEGs and 4 DEGs in DRG and SCDH were related to the Wnt pathway, respectively. Then, we performed gene ontology analysis by the Panther Classification System database system to enrich the pathways involved in proteins encoded by DEGs in DRG and SCDH and found that 4 DEGs in DRG and 1 DEG in SCDH related to the Wnt pathway were screened out. After removing the duplicated genes, we screened out 12 and 4 genes in DRG and SCDH, respectively (Table 1).

### 3.3. Activation of Wnt/*β*-Catenin Induced Cytokines in Both DRG and SCDH in CCD

DRG and SCDH changes caused by nerve injury are critical for the generation and persistence of NP. We addressed whether the Wnt/*β*-catenin pathway in DRG and SCDH in CCD rats has changed. Active *β*-catenin is a critical protein in this pathway and whether it undergoes nuclear translocation reflects whether Wnt/*β*-catenin is activated. Therefore, we detected the level of active *β*-catenin by western blot and nuclear translocation of active *β*-catenin by immunofluorescence. As is shown in western blot results, the compression of DRG resulted in a rapid rise in the expression of active *β*-catenin in DRG (Figure 2(a)) and SCDH (Figure 2(b)) (within 1 day) and increased continuously (*P* < 0.05). Both reached a peak of expression in 7-14 days and then gradually declined. Additionally, immunofluorescence experiments showed that after 7 days of modeling, a large number of active *β*-catenin positive stains (red) were seen on the left DRG (Figure 2(c)) and SCDH (Figure 2(d)) in the CCD model rats, and the positive staining was stronger than that in the sham group. Colocalization of active *β*-catenin (red) and DAPI (blue) showed that the expression of active *β*-catenin in the nucleus rose in CCD rats. To further explore the potential mechanism of the Wnt/*β*-catenin pathway affecting NP, we detected the expression levels of TNF-*α* and IL-18, which are the proinflammatory cytokines in serum by ELISA. The results showed that the level of TNF-*α* and IL-18 in rat serum increased significantly on the first day (*P* < 0.0001) and reached the peak at 7 days, and then, TNF-*α* gradually decreased, while IL-18 remained at a stable level until postoperative 28 days (*P* < 0.0001) (Figures 2(e) and 2(f)). In addition, the results of Spearman correlation coefficient analysis showed that the levels of TNF-*α* (Spearman correlation coefficient: -0.829, *P* < 0.05) and IL-18 (Spearman correlation coefficient: -0.943, *P* < 0.01) were negatively correlated with MWT after CCD surgery, which meant that the higher the levels of TNF-*α* and IL-18, the more obvious the pain in rats, and vice versa, the pain in rats was relieved.

### 3.4. Blocking the Wnt/*β*-Catenin Pathway Suppressed the Cytokines for the Development of Allodynia in CCD

Next, to investigate whether the Wnt/*β*-catenin pathway makes a critical impact on the pathogenesis and maintenance of neuropathology, we performed intraperitoneal injection of XAV939, a Wnt/*β*-catenin pathway inhibitor, in CCD rats for seven consecutive days and tested behavioral changes daily (timeline is shown in Figure 3(a)). Our results showed that XAV939 can alleviate NP after CCD. At 5-7 days of injection, the MWT of the hind paw significantly increased (*P* < 0.0001) (Figure 3(b)). Furthermore, we confirmed that XAV939 did inhibit the Wnt/*β*-catenin pathway via western blot and immunofluorescence experiments. The results showed that XAV939 did inhibit active *β*-catenin accumulation in DRG and SCDH (Figures 3(c) and 3(d)). Correspondingly, the expression of TNF-*α* and IL-18 was also significantly reduced (Figures 3(e) and 3(f)) when we inhibited this pathway by XAV939 (*P* < 0.0001). The results above demonstrated that the activation of the Wnt/*β*-catenin pathway affected the persistence of NP and the expression of TNF-*α* and IL-18 was regulated by the activation of the Wnt/*β*-catenin pathway after CCD.

## 4. Discussion

LBP is one of the most common pains in the clinic. Mechanical compression and chemical stimulation of DRG may lead to ischemia, edema, and degeneration of DRG and eventually leading to the development of allodynia [29, 30]. However, the specific mechanism of NP is still unclear. Our study brings a key role for the Wnt/*β*-catenin pathway in the induction and continuation of NP following chronic compression of nerve to light. The main findings can be attributed to the following three aspects: (1) chronic nerve compression led to changes in the expression of multiple Wnt pathway-related genes and rapid and sustained activation of the Wnt/*β*-catenin pathway in DRG and SCDH; (2) inhibition of activation of the Wnt/*β*-catenin pathway alleviated allodynia induced by chronic nerve compression; (3) CCD led to elevating the level of TNF-*α* and IL-18. TNF-*α* and IL-18 levels were significantly correlated with MWT, while blocking the Wnt/*β*-catenin pathway decreased the levels of TNF-*α* and IL-18.

Wnt is very important for various development processes. The Wnt pathway was first revealed by scientists in the development of Drosophila [31] and is a key signaling pathway regulating neuronal development, neuronal polarization, synaptic plasticity changes, and directional growth of axons and dendrites [32, 33]. Previous studies have revealed that the Wnt/*β*-catenin pathway is activated in SCDH in several NP models, such as CCI and PSL [15, 18]. Besides, studies showed that the levels of multiple inflammatory factors increased in the serum of clinical patients including IL-18 and TNF-*α* [34, 35] and pain intensity correlated with the levels of inflammatory factors [36]. The reason for choosing TNF-*α* and IL-18 among many elevated inflammatory factors was that these two inflammatory factors were not only closely related to pain, but also target genes closely downstream of the Wnt/*β*-catenin pathway [15]. These studies suggested that the Wnt/*β*-catenin pathway makes an important impact on the development and progression of NP, and the activation of this pathway may participate in the pathogenesis of NP by regulating the transcription of TNF-*α* and IL-18, which are closely related to pain.

Our study found that active *β*-catenin was immediately and continuously upregulated in DRG and SCDH in the CCD model, and immunofluorescence results confirmed the translocation of active *β*-catenin into the nucleus, which can more intuitively observe the localization of active *β*-catenin protein in cells and more powerful than the extraction of active *β*-catenin protein in the nucleus to prove the nuclear translocation of active *β*-catenin protein and the activation of the Wnt/*β*-catenin pathway. This suggested the activation of the Wnt/*β*-catenin pathway lasted for a long time, which was consistent with previous studies in other models [15, 18]. Additionally, we found that the levels of TNF-*α* and IL-18, which are closely related to NP, were considerably raised in the serum of CCD rats; however, after inhibiting this pathway, the levels of TNF-*α* and IL-18 correspondingly decreased. Moreover, the levels of TNF-*α* and IL-18 were significantly correlated with the allodynia time of CCD rats. These results implicated blocking the Wnt/*β*-catenin pathway can inhibit NP by decreasing the level of IL-18 and TNF-*α*. These results revealed that the Wnt/*β*-catenin pathway takes part in the development of NP after compression of DRG and is likely to affect NP by regulating the transcription of downstream inflammatory factors. Mechanisms underlying contributions of the Wnt pathway to neuropathic pain are summarized in Figure 4.

What is more, many scholars have conducted extensive research on the mechanism of NP, and it is believed that NP is caused by peripheral sensitization and central sensitization [37, 38]. Peripheral sensitization refers to an increase in the excitatory persistent abnormalities of primary afferent neurons, resulting in increased pain signal production [39]; central sensitization refers to the plasticity change of synaptic in SCDH, and the long-term potential (LTP) of synaptic transmission efficiency in the pain transmission pathway [40]. Studies have shown that the Wnt pathway can regulate neuronal firing activity [41, 42] and enhance synaptic plasticity by promoting synapse formation such as in the hippocampus [43, 44]. Therefore, we conjectured that the Wnt/*β*-catenin pathway may also induce peripheral sensitization and central sensitization by increasing neuronal excitability in DRG and increasing synaptic strength in SCDH, thereby affecting the progression of NP.

In summary, our research brings a pivotal role for the Wnt/*β*-catenin pathway in the production and persistence of NP after chronic compression of DRG to light. Additionally, the Wnt/*β*-catenin pathway may induce NP through modulating the levels of TNF-*α* and IL-18. Moreover, it provides new targets and new ideas for the treatment of nerve compression diseases including LFS and LDH and may also be one of the ways for some drugs and biological treatments such as stem cells to exert analgesic effect.

## Figures and Tables

**Figure 1:** The CCD model and the development of mechanical allodynia after establishment of the CCD. (a) Schematic diagram of CCD generated by inserting stainless steel rod into L4 and L5 intervertebral foramina of rats. (b) CCD-induced mechanical allodynia is manifested by a reduction of MWT. Bars represent group means ± SD, *n* = 12 per group. Two-way ANOVA, ^∗∗∗∗^*P* < 0.0001 versus sham.

**Figure 2:** Expression and nuclear translocation of active *β*-catenin protein in DRG and SCDH and the levels of TNF-*α* and IL-18 in serum after CCD. Western blot showing the expression of active *β*-catenin in (a) DRG and (b) SCDH at different time points. The expression of active *β*-catenin (red) and its transport of the superficial (c) DRG and (d) SCDH into the nucleus (DAPI). Arrows indicate some of the nuclear transport of active *β*-catenin. Tissues were collected on CCD day 7. The sections were imaged with a (c) fluorescence microscope and a (d) confocal microscope. Original magnification, scale bars: 20 *μ*m. ELISA displaying the levels of (e) TNF-*α* and (f) IL-18 in rat serum at different time points after CCD (*n* = 6). Serum was collected on CCD day 7. Bars represent group means ± SD, *n* = 5. One-way ANOVA, ^∗^*P* < 0.05, ^∗∗^*P* < 0.01, ^∗∗∗^*P* < 0.001, and ^∗∗∗∗^*P* < 0.0001 versus sham.

**Figure 3:** Intraperitoneal injection of XAV939 attenuated mechanical allodynia and decreased TNF-*α* and IL-18 levels in serum after CCD. (a) Schematic time course for acclimation, CCD surgery, intraperitoneal injection of XAV939, behavioral testing, and sacrifice. (b) MWT measured on 0, 1, 3, 5, and 7 days after CCD treatment (*n* = 9). Two-way ANOVA. Western blot showing active *β*-catenin expression in (c) DRG and (d) SCDH (*n* = 6). ELISA showing the expression of (e) TNF-*α* and (f) IL-18 in the serum of rats after intraperitoneal injection of XAV939 (*n* = 6). Serum was collected at different time points after CCD. One-way ANOVA. Bars represent group means ± SD. ^####^*P* < 0.0001, CCD+vehicle versus sham; ^∗∗∗∗^*P* < 0.0001, CCD+XAV939 versus CCD+vehicle.

**Figure 4:** Schematic illustration of the relationship between the Wnt/*β*-catenin pathway and neuropathic pain. The relationship between the Wnt/*β*-catenin pathway and neuropathic pain in the CCD model was possibly that CCD surgery caused activation of the Wnt/*β*-catenin pathway; then, active *β*-catenin accumulated in the cytoplasm and translocated into the nucleus. Subsequently, the transcription of the target genes TNF-*α* and IL-18 increased, leading to neuropathic pain finally, while the Wnt/*β*-catenin inhibitor XAV939 can suppress this process, relieving CCD-induced neuropathic pain.

**Table 1:** DEGs related to Wnt pathway in DRG and SCDH of rats 28 days after CCD.

Gene symbol	Description	log_2_ fold change	Direction	*P* value
*DRG*				
Npy	Neuropeptide Y	3.9458	↑	<0.001
Runx2	Runt-related transcription factor 2	1.3276	↑	<0.001
Cthrc1	Collagen triple helix repeat containing 1	2.3058	↑	<0.0001
Draxin	Dorsal inhibitory axon guidance protein	2.3726	↑	<0.01
Cpz	Carboxypeptidase Z	-1.2635	↓	<0.01
Kb15	Type II keratin Kb15	-1.9539	↓	<0.05
Tnn	Tenascin N	2.6944	↑	<0.01
Amer2	APC membrane recruitment protein 2	-1.8238	↓	<0.01
Pcdh20	Protocadherin 20	1.7709	↑	<0.001
Pcdh8	Protocadherin 8	-1.1441	↓	<0.01
Myh3	Myosin heavy chain 3	-1.9875	↓	<0.05
Gnb3	G protein subunit beta 3	-1.0005	↓	<0.05

*SCDH*				
Mcc	Colorectal mutant cancer protein	-2.2131	↓	<0.05
Egf	Epidermal growth factor	1.1111	↑	<0.0001
Cdh1	Cadherin 1	1.7580	↑	<0.05
Plekha4	Pleckstrin homology domain containing A4	1.4888	↑	<0.001

## Data Availability

GraphPad Prism 7.0 software (GraphPad Software Inc., CA, USA) and SPSS 20.0 software (IBM Corporation, NY, USA) were applied to analyze all data.
